# NORAD Promotes the Viability, Migration, and Phenotypic Switch of Human Vascular Smooth Muscle Cells during Aortic Dissection via LIN28B-Mediated TGF-*β* Promotion and Subsequent Enhanced Glycolysis

This article has been retracted.

**DOI:** 10.1155/2022/5333928

**Published:** 2022-08-06

**Authors:** Shi-bo Xia, Zhuang-bo Tian, Wenbo Zhang, Hao Zhang

**Affiliations:** ^1^Department of Vascular Surgery, Changhai Hospital, Second (Navy) Military Medical University, Shanghai 200433, China; ^2^Department of Interventional Vascular Surgery, Hunan Provincial People's Hospital/The First Affiliated Hospital of Hunan Normal University, Changsha, Hunan 410005, China; ^3^Department of Cardiac Surgery, Beijing Anzhen Hospital, Capital Medical University, Beijing 100029, China

## Abstract

Glucose metabolism reprogramming is an important reason for the functional remodeling, growth, and migration of vascular smooth muscle cells (VSMCs). It is also an important basis for the occurrence and development of aortic dissection (AD), but the specific regulatory factors are not clear. Noncoding RNA activated by DNA damage (NORAD) is dysfunctional in many diseases, but the role of NORAD in AD etiology is unclear. We first established a vascular remodeling cell model of AD, and the expression of NORAD in VSMCs was significantly increased. Functional experiments showed that inhibition of NORAD could downregulate the proliferation and migration of VSMCs. Meanwhile, silencing NORAD could also inhibit the flux of glycolysis, suggesting that NORAD may aggravate AD by promoting glycolysis. In addition, mechanism studies have shown that NORAD can exert VSMCs-regulating function by recruiting LIN28B to bind to TGF-*β* mRNA, which subsequently facilitates the expression of TGF-*β*1 (transforming growth factor *β*1). The recovery experiment also showed that overexpression of TGF-*β* could reverse the inhibitory effect of NORAD knockdown on VSMCs in terms of proliferation, migration, and glycolysis. Collectively, these results indicated that the NORAD/LIN28B/TGF-*β* axis promoted cell proliferation and migration through regulating aerobic glycolysis in VSMCs. Therefore, NORAD may regulate the occurrence of AD by affecting the reprogramming of glucose metabolism, and NORAD can be recognized as a good target for VSMC phenotypic intervention and AD treatment.

## 1. Introduction

Aortic dissection (AD) is a kind of cardiovascular disease, which is fatal and seriously affects the prognosis of patients. AD can often show symptoms of chest pain. When the arterial membrane is torn or bleeding due to atherosclerosis or trauma, it can lead to partial separation of the arterial wall, resulting in AD [1]. AD is characterized by vascular occlusion and hyperresponsiveness, in which vascular remodeling plays a central role [2]. At present, the etiology of AD is unknown, but many determinants, including genetic factors, environmental pollution, and parental and baby nutritional condition have a role in the pathophysiology of AD [3, 4]. The functional abnormality of VSMC is an important mechanism of AD [5]. For example, platelet-derived growth factor (PDGF) enhances hematal restructuring in Alzheimer's disease by causing extreme VSMC multiplication [6]. Therefore, it is generally believed that ASM cell proliferation is related to the severities of AD. As VSMC not only is seen as the primary essential constituent of the vessel but also regulates the function of the vascular, how to inhibit the proliferation of VSMCs to control vascular remodeling has become one of the bases for the treatment of AD [7]. However, the regulatory factors of VSMC proliferation remain unclear.

VSMC remodeling, including increased growth and accelerated migration, is still a clear sign of bronchial remodeling in AD. TGF-1 (transforming growth factor *β*1) is an important cytokine, which can promote the migration of immune cytokines and vascular remodeling in AD [8]. Activated TGF-1 levels in bronchoalveolar lavage fluid were shown to be increased in AD [9]. Bronchodilators and antiphlogistic medicine drugs are the only standard therapy for AD [10]. As a result, emerging treatment approaches targeting VSMC reconfiguration will be critical in AD treatment.

Metabolic reprogramming of cells under pathological conditions is a typical feature of the occurrence and progression of the disease including AD [11], in which glucose metabolic reprogramming, in terms of glycolysis, has been studied most frequently. During the occurrence of AD, VSMCs will also undergo metabolic reprogramming, which is beneficial to the enhancement of cell activity and invasiveness and eventually leads to vascular remodeling [12]. However, the relationship between glycolysis and vascular remodeling and the upstream regulatory factors remain to be determined.

Long-chain noncoding RNA (lncRNA) is a RNA molecule with a length of more than 200 bp but does not have the ability to encode a protein. There is growing evidence that lncRNA plays a role in the origin and progression of many cancers, especially AD. It has also been shown to play an important role in VSMC, thus affecting the AD curriculum. For example, lncRNA BCYRN1 increases the growth and metastasis of rat VSMC by overexpressing transient receptor potentials [13]. GAS5 enhances the growth of VSMC in AD through modulating the miR-10a/BDNF signaling pathway [14]. As a result, a clearer understanding of the biological processes regulated by lncRNA in AD can aid diagnoses and pave the opportunities for sustainable progress of effective and new therapy options for the disease.

We speculate that the level of noncoding RNA activated by DNA damage (NORAD) in the noncoding region activated by DNA damage in VSMC is increased, NORAD gene knockout can inhibit the proliferation and migration of VSMC, and NORAD may regulate the occurrence of AD through reprogramming that affects glucose metabolism, so we carried out this study.

## 2. Materials and Methods

### 2.1. Vascular Smooth Muscle Cell (VSMC) Isolation and Culture

As has been publicly confirmed, VSMC in the AD rat model has been identified and standardized. After the rats were killed under anesthesia, the trachea was removed, and the epithelial fibrous tissue was removed. The remaining tissue was stored in PBS and degraded by various enzymes at 37°C. After digestion, the free VSMC was centrifuged and incubated with RPMI-1640 and 10% fetal bovine serum (FBS).

### 2.2. Cell Transfection

shRNA of lnc-NORAD and control (sh-NC) was bought from Novoprotein Technology (Shanghai, China). The entire cDNA of TGF-*β* was introduced into the pcDNA3.1 template (Takara, Otsu, Japan). Following incubation for 24 h, VSMC was transduced by sh-NORAD or sh-NC solely or in combination with pcDNA3.1/TGF-*β* or pcDNA3.1 vector as needed. The cells were transfected with Lipofectamine 3000 (Life Technologies, US) for two days based on the production's instructions.

### 2.3. Quantitative Real-Time PCR (qRT-PCR)

Following extraction from cells by the RNAiso Plus Kit (Takara, Japan) according to the production's guidelines, RNA was totally synthesized utilizing the GoScript Reverse Transcription System (Promega, USA). The SYBR Green PCR Kit (Takara, Japan) was applied to the amplification in the RT-PCR assay. GAPDH was employed as an internal reference.

### 2.4. Cell Viability/Proliferation Assays

Cell growth was examined via VSMC viability and proliferation, respectively. Cells were planted at a density of 1.5 × 10^3^ into the 96-well plate. Then, cell viability was tested utilizing the MTT Assay Kit (Abcam, US). The cellular proliferation was performed by the BrdU Cell Proliferation ELISA Kit (Abcam, US) according to the protocols.

### 2.5. Transwell Assay

Matrigel was applied to detect the capacity of cells to migrate (Millipore, Billerica, MA, US). VSMCs (1 × 10^5^) resuspended in 100 ml of DMEM were introduced to the upper chamber, while 600 ml of DMEM with 10% FBS was given to the bottom chamber. VSMCs that had moved into the bottom chamber were fixed with 4% formalin solution, dyed with 0.5 percent crystal violet, and quantified using optical microscopy (Leica, Germany).

### 2.6. RNA Immunoprecipitation (RIP) Assay

The RNA Immunoprecipitation (RIP) Kit (Bersin Bio) was used in the RIP assays. RIP lysate was used to obtain cell extracts, which were then combined to magnetic beads and antibody against EIF4A3 (Sigma-Aldrich). The secondary antibody was Anti-IgG (Sigma-Aldrich). The isolated coprecipitation RNA was submitted to the qRT-PCR assay.

### 2.7. Actinomycin D Treatment

After transfection, 2 mg/ml Actinomycin D (Abcam, US) was put into the medium to stop the transcriptional process. The residual mRNA was measured utilizing qRT-PCR following administration with Actinomycin D for various time points.

### 2.8. Subcellular Fractionation Assay

To isolate RNA in the nucleoplasm, the PARIS Kit (Life Technologies, CA) was used. In a word, samples were extracted, digested on freezing, and then centrifuged at 12,000g for 3 minutes. U6 and GAPDH were used as nuclei reference and cytoplasmic reference, respectively. The precipitate was tested for cytoplasmic RNA, and the nuclei pellet was applied to identify nuclei RNA.

### 2.9. Statistical Analysis

All data collection was carried out with SPSS 23.0, and all experimental findings were presented as the mean ± SD. All the data conform to the normal distribution, and the *t*-test was used to analyze the statistical differences between the two groups. One-way ANOVA was used to examine comparisons between three or more groups. In order to have statistical significance, the *P* value cut-off selection is 0.05.

## 3. Results

### 3.1. lncRNA NORAD Is Upregulated in the VSMCs of Rat AD Models and Promotes the VSMC Proliferation and Migration

Firstly, we constructed the rat AD model and extracted the VSMCs from the rat vascular. RT-PCR showed that lncRNA NORAD was significantly upregulated in the VSMCs of AD compared to control, and there was a significant difference between the groups (*P* < 0.05) (Figure 1(a)). Thus, in order to delineate the function of NORAD for the VSMC phenotype, silencing of NORAD was constructed using shRNA plasmid transfection, and there was a significant difference between the groups (*P* < 0.05) (Figure 1(b)). The CCK-8 assay indicated that silencing of NORAD inhibited the proliferation ability of VSMCs, and there was a significant difference between the groups (*P* < 0.05) (Figure 1(c)). In addition, cross-well experiments were used to examine the effect of NORAD on VSMC migration. The results show that the reduction of NORAD greatly reduces the ability of VSMC migration, and there was a significant difference between the groups (*P* < 0.05) (Figure 1(d)). Therefore, the above results suggest that the upregulated lncRNA NORAD promotes the proliferation and migration of VSMCs.

### 3.2. NORAD Knockdown Attenuates Aerobic Glycolysis in VSMCs

Enhanced aerobic glycolysis is a common feature of many diseases, including AD. Considering the possible relationship between aerobic glycolysis and AD, we investigated whether NORAD regulated aerobic glycolysis in VSMCs. At the beginning, knocked down NORAD markedly decreased glucose intake of VSMCs (Figure 2(a)), lactic (Figure 2(b)), and ATP generations (Figure 2(c)), and there was a significant difference between the groups (*P* < 0.05). In addition, NORAD knockdown in VSMCs resulted in a lower extracellular acidification rate (ECAR), which is a measure of cellular total glycolysis flux, and there was a significant difference between the groups (*P* < 0.05) (Figure 2(d)). Moreover, the oxygen consumption rate (OCR), an index of mitochondrial respiration, was significantly increased in NORAD knockdown VSMCs, and there was a significant difference between the groups (*P* < 0.05) (Figure 2(e)). Collectively, these results strongly suggested that NORAD was involved in the aerobic glycolysis process in VSMCs.

### 3.3. NORAD Recruited LIN28B to Stabilize TGF-*β* mRNA

The localization of lncRNA in cells is significantly related to its function. Based on this, we first analyzed the subcellular localization of NORAD and NORAD mostly generated in the plasma, according to intracellular fraction studies, suggesting that NORAD may take a regulated part in the transcription or posttranscription of the target gene, and there was a significant difference between the groups (*P* < 0.05) (Figure 3(a)). In order to identify the target gene of NORAD, we detected several important targets involved in the regulation of cellular growth. The data suggested that after the downregulation of NORAD, only the mRNA level of TGF-*β* displayed greatly affected. Meanwhile, the western blot also showed that the protein expression of TGF-*β* was significantly decreased while downregulating NORAD. The above results suggest that TGF-*β* may be the regulatory target gene of NORAD. lncRNA regulates the stability of downstream target genes through RNA-binding proteins, which is an important way for lncRNA to contribute to a regulatory role. To identify the RNA-binding proteins that interact with lncRNA, we use the RIP test to verify the proteins that interact with lncRNA. The results show that LIN28B may be a RNA-binding protein interacting with lncRNA, and there was a significant difference between the groups (*P* < 0.05) (Figures 3(b)–3(d)). In addition, RIP experiments also confirmed the interaction between LIN28B and TGF-*β* mRNAs, which can be eliminated by NORAD knockdown. As expected, NORAD knockdown induces high expression of LIN28B, resulting in TGF-*β* mRNA stability and TGF-*β* stability rebound, and there was a significant difference between the groups (*P* < 0.05) (Figure 3(f)). All these data show that NORAD affects the expression of TGF-*β* by participating in LIN28B, thus improving the stability of TGF-mRNA.

### 3.4. NORAD Facilitates VSMC Growth and Migration via NORAD/LIN28B/TGF-*β* Axis

NORAD was used in rescuing tests to see if TGF-*β* impacted the growth and metastasis of VSMCs. While TGF-*β* was abundantly expressed, cell viability was suppressed by suppression of NORAD, as seen in Figure 4(a), and there was a significant difference between the groups (*P* < 0.05). It was claimed that ectopic TGF-*β* expression prevented the NORAD knockdown-induced decrease in migration, and there was a significant difference between the groups (*P* < 0.05) (Figure 4(b)). To summarize, NORAD induced AD-promoting characteristics in VSMCs through TGF-*β* regulation. Moreover, TGF-*β* upregulation reversed the NORAD knockdown-induced reduction of glucose utilization and lactic generation, and there was a significant difference between the groups (*P* < 0.05) (Figures 4(c) and 4(d)). In addition, according to ECAR and OCR analysis, upregulation of TGF-*β* partially compensates for the damage of glycolysis caused by NORAD silencing, and there was a significant difference between the groups (*P* < 0.05) (Figures 4(e) and 4(f)). In summary, these results suggest that the NORAD/LIN28B/TGF-*β* axis promotes cell proliferation and migration by regulating aerobic glycolysis in VSMC.

## 4. Discussion

This study identified that the noncoding RNA activated by DNA damage (NORAD) level in VSMC was obviously increased, and NORAD knockdown could impede the proliferation and migration of VSMCs; meanwhile, the silence of NORAD could also inhibit glycolysis. In addition, mechanism studies have shown that NORAD can exert VSMCs-regulating function by recruiting LIN28B to bind to TGF-*β* mRNA. These results indicated that the NORAD/LIN28B/TGF-*β* axis promoted cell proliferation and migration through regulating aerobic glycolysis in VSMCs. Therefore, NORAD may regulate the occurrence of AD through reprogramming that affects glucose metabolism, and NORAD can be used as a good target for VSMC phenotypic intervention and AD therapy.

That being said, VSMC performed important parts in the pathogenesis and development of AD, according to mounting evidence [15, 16]. Blood flow redistribution can be observed in AD because the intima of the artery is torn and impacted by the blood flow, resulting in different vascular cavities, which is a sign of AD. Arterial intimal tear leads to structural changes in blood vessels, which affects the thickness of the arterial wall, the elasticity of blood vessels, and the width of the vascular lumen [9, 17]. In particular, the blood model in AD is likely to be a sign of the excessive quality of VSMC, which is related to the growth and migration of VSMC [14]. In addition, VSMC can produce inflammatory mediators and release extracellular matrix proteins, all of which are associated with cell growth, migration, and death [18]. Accordingly, the blood wall thickness is caused by downregulation of VSMC differentiation and growth, which leads to vascular remodeling in AD [19]. As a result, it is critical to continue research into the biomolecular mechanisms underpinning VSMC growth and metastasis in AD. Increasing evidence suggests that lncRNA plays a role in respiratory illness biology through epigenetic modifications and genome imprints, increased expression, and epigenetic control [20]. For instance, lncRNA-GAS5 has been revealed to behave as deception in the regulation of glucocorticoid resistance [14]. lncRNA-PVT1 was found to be increased in individuals with corticosteroid-resistant severe AD, suggesting that it may be implicated in glucocorticoid-resistant modulation [21]. Recently, NORAD's role in pathological disorders has been emphasized [22]. NORAD is upregulated in a variety of cancers and is linked to prognosis [23]. Elevated levels of NORAD have been commonly investigated in lung cancer, which is linked to negative outcomes [24]. However, the mechanism of NORAD in the respiratory system especially in AD and vascular remodeling is yet to be elucidated. We observed that NORAD was upregulated significantly in VSMCs after AD. Concomitantly, we showed that the knockdown of NORAD VSMCs attenuated cell proliferation and migration. Considering that cellular growth is involved in vascular rebuilding. NORAD probably have a crucial function in children's AD.

Previous research has shown that lncRNA can engage RBPs to modulate the mRNA stabilization of their target genes [25]. The RBPs that potentially interact with NORAD were discovered using RIP analysis in the current investigation. LIN28B, a major element of the exon junction complexes, can limit TGF-*β* mRNA degradation and modulate the transcription at the genomic and epigenetic levels among many other things. This research investigates and identifies the epigenetic regulation of NORAD on the VSMC via the RNA-binding protein regulation mechanism. This pathway of RNA-binding protein provides an excellent regulating manner for the lncRNA. Via this pathway, NORAD could promote the proliferation and migration of VSMC in the AD. Then, we carried out a chain of measurements and observed that the inhibitory effect of NORAD knockdown on VSMC growth and migration was greatly changed via TGF-*β* high expression. This finding implies that the NORAD knockdown-induced reduction of VSMC growth and invasion needs TGF-*β* activity. According to existing research, a variety of biosynthetic processes may play a key role in the innate immune system of AD [26]. Solving key metabolic catalysts or sensors to restore normal metabolism may provide new treatment strategies for respiratory problems and dysfunction [27]. Gluconeogenetic activation is usually related to the decrease of OXPHOS and the transition to biochemical processes. It is the initial activity of various cell growth, development, migration, differentiation, and activation of inflammation, making it a promising therapeutic target for inflammatory diseases [28]. What is particularly noteworthy is that our research shows that knocked down NORAD gene can remarkably reduce the glycolysis level of VSMCs in terms of glucose uptake ability and ATP production ability, accompanied by the switching of ECAR to OCR metabolic modes. These results indicated that the NORAD/LIN28B/TGF-*β* axis promoted cell proliferation and migration through regulating aerobic glycolysis in VSMCs. There are some limitations to this study. First, the sample size of this study is not large, and it is a single-center study, so bias is inevitable. In future research, we will carry out multicenter, large-sample prospective studies, or more valuable conclusions can be drawn.

Ultimately, this study identified potential biological pathways for vascular remodeling controlled by VSMC. The upregulation of NORAD promotes the proliferation and migration of VSMC through posttranscriptional regulation of TGF-*β*. All the results are helpful to reveal the biochemical pathways associated with VSMC-related vascular remodeling, thus providing new potential biomarkers for diagnosis or treatment.

## Figures and Tables

**Figure 1:** NORAD is upregulated in VSMCs of rat AD models and promotes the VSMC growth and migration. (a) NORAD level in AD VSMCs and VSMCs controls was examined by qRT-PCR. (b) The efficiency of NORAD knockdown in VSMCs was verified by qRT-PCR. (c) The impact of NORAD silencing on VSMC efficiency was assessed by the CCK-8 test. (d) The impacts of NORAD silence on the migration of VSMCs were determined using the transwell assay. Data were represented as the mean ± SD. ^∗^*P* < 0.05 was shown in comparison to the negative control.

**Figure 2:** NORAD knockdown dampens the aerobic glycolysis in VSMCs. (a) Glucose intake of VSMCs was determined. (b) Lactate production of VSMCs was determined. (c) ATP of VSMCs was determined. (d, e) ECAR of VSMCs was studied. Data were represented as the mean ± SD. ^∗^*P* < 0.05 was shown in comparison to the negative control.

**Figure 3:** NORAD recruited LIN28B to stabilize TGF-*β* mRNA. (a) Subcellular fractionation test was performed to confirm the nuclear-cytoplasmic fractionation of NORAD in VSMCs. (b) Effect of NORAD silence on the mRNA expression of PDGF, VEGF, FGF, and TGF-*β*. (c) Effect of NORAD silence on the protein TGF-*β* level. (d) The interreaction of NORAD and RNA-binding protein was verified by RIP. (e) The impact of NORAD silencing on the complex of LIN28B to TGF-*β* was evaluated by the RIP assay. (f) The mRNA stabilization of TGF-*β* was detected by qRT-PCR. Data were presented as the mean ± SD. ^∗^*P* < 0.05 was shown in comparison to the negative control.

**Figure 4:** NORAD facilitates VSMC growth and migration via NORAD/LIN28B/TGF-*β* axis. (a) TGF-*β* high expression partially corrected the antagonistic impact of NORAD silencing upon the CCK-8 assay of VSMCs. (b) TGF-*β* overexpression partly reversed the effects of NORAD knockdown on migration of VSMCs. (c, d) The impact of NORAD silencing on the suppression of glucose intake and lactate generation in VSMCs could be rescued by TGF-*β* overexpression. (e, f) TGF-*β* overexpression could rescue the antagonistic impact of NORAD silencing on the glycolytic process in VSMCs, as reflected by ECAR and OCR analysis. Data were represented as the mean ± SD. ^∗^*P* < 0.05 was shown in comparison to the negative control. ^#^*P* < 0.05 was shown in comparison to the sh-NORAD with the negative control.

## Data Availability

The datasets used and analyzed during the current study are available from the corresponding author upon reasonable request.
